RETRACTED

# Effects of Electroacupuncture with Different Waveforms on Chronic Prostatitis/Chronic Pelvic Pain Syndromes: A Randomized Controlled Trial

**DOI:** 10.1155/2022/6866000

**Published:** 2022-07-13

**Authors:** Zhihao Li, Juan Liu, Peng Liu, Yahui Zhang, Wenjun Han

**Affiliations:** ^1^Shanghai University of Traditional Chinese Medicine, 1200 Cailun Road, Pudong New Area, Shanghai 201203, China; ^2^The Seventh People's Hospital Affiliated to Shanghai University of Traditional Chinese Medicine, 358 Daotong Road, Pudong New Area, Shanghai 200137, China

## Abstract

Chronic prostatitis/chronic pelvic pain syndrome (CP/CPPS) is a common disorder in adult men. Evidence has demonstrated that acupuncture is effective for treating CP/CPPS. Electroacupuncture (EA) is a combination of traditional acupuncture and electrical stimulation, and the waveform is one of the key factors influencing EA effects. Different waveforms contain different stimulating parameters, thus generating different effects. However, the effects of different waveforms of EA on CP/CPPS remain unclear and there is no recommended standard for the application of EA waveforms. At the same time, the waveform prescription of CP/CPPS is also different, so exploring the influence of different waveforms on CP/CPPS patients will also provide a certain treatment basis for clinical treatment. A total of 108 eligible patients were recruited from the Seventh People's Hospital affiliated to the Shanghai University of Traditional Chinese Medicine from March 18, 2021, to January 31, 2022, according to inclusion and exclusion criteria. All subjects were randomly divided into three groups (continuous wave 4 Hz, continuous wave 20 Hz, and extended wave 4/20 Hz) in a ratio of 1 : 1 : 1. Patients in all three groups were treated for the same duration of 20 minutes, with intervention twice a week for 4 weeks. The changes in chronic prostatitis index (NIH-CPSI), erectile function index 5 (IIEF-5), Hospital Anxiety and Depression Scale (HADS), and NIH-CPSI response rate in three groups were compared after the intervention, and the occurrence of adverse events in patients during treatment was observed. After 4 weeks of treatment, the CP/CPPS response rates were 66.7%, 62.5%, and 88.2% in the 4 Hz, 20 Hz, and 4/20 Hz groups, respectively. The reaction rate of CP / CPPS in 4 / 20 Hz group was higher than that in 4 Hz group and 20 Hz group. (*P* < 0.05). During treatment, the difference between NIH-CPSI scores between 4 Hz and 4/20 Hz was insignificant (*P* > 0.05). NIH-CPSI scores were lower in the 4/20 Hz group than in the 4 Hz and 20 Hz groups (*P* < 0.05). After treatment, there was no significant difference in the pain and discomfort subscales (*P* > 0.05) between the 4 Hz and 20 Hz groups and there were significantly lower pain and discomfort scores in the 4/20 Hz group (*P* < 0.05) compared to the 4 Hz and 20 Hz groups. There was no significant difference in the reduction of urination symptoms and quality of life among the three groups (*P* > 0.05). Compared with before treatment, IIEF-5 scores of the three groups were improved (*P* < 0.05). After treatment, there was no significant difference between the IIEF-5 scores in 4 Hz and 20 Hz (*P* > 0.05), while the IIEF-5 score in 4/20 Hz was significantly higher than that in 4 Hz and 20 Hz, and the change was significant (*P* < 0.05). The HADS scores decreased in all the three groups (*P* < 0.05), but there was no significant difference in HADS scores between the three groups (*P* > 0.05). Adverse events were mild and transient, and no serious adverse events occurred in each group. Both the expansive and continuous waveforms of EA can effectively alleviate symptoms such as prostatitis, erectile dysfunction, anxiety, and depression in patients with CP/CPPS. Expansion waves are superior to continuous waves in improving erectile function and pain symptoms in chronic prostatitis and can be used as a preferred waveform for the treatment of CP/CPPS. *Trial Registration.* This trial is registered with Chinese Clinical Trial Registry, ChiCTR2100044418.

RETRACTED

## 1. Introduction

Chronic prostatitis/chronic pelvic pain syndrome (CP/CPPS) is a common disorder in adult men. The main symptoms of CP/CPPS include low abdominal pain and abnormal urination, such as frequent urination, urgent urination, and dysuria, which have a considerable impact on the life and health of patients [1]. Nearly half of the men will be affected by prostatitis in their lives [2], and CP/CPPS accounts for 90%–95% of all diagnoses of prostatitis [3]. The prevalence rate ranges from 2.2% to 9.7% and 4.5% in China [4, 5].

Although its incidence is high, its pathogenesis is still unknown. Thus, the current treatment is still mainly symptomatic treatment, such as relieving pain and discomfort and improving urination symptoms and quality of life [6]. Common drugs include *α*-adrenergic receptor blockers, antibiotics, nonsteroidal antiinflammatory drugs, and 5-*α* reductase inhibitors [6]. However, these medicines have some side effects, such as hypotension, gastrointestinal dysfunction, and hypolibido [7]. In addition, several studies indicated that antibiotics and *α*-adrenergic receptor blockers or NSAIDs did not show ideal effects on CP/CPPS [8, 9], which leads to substantial psychological and economic burdens among patients [10, 11]. Thus, safe, economical, and effective measures are needed.

RETRACTED

Acupuncture has a long history and has been widely used in clinical practice due to its advantages of safety and convenience. Acupuncture is an effective intervention for CP/CPPS, especially in relieving pain symptoms and improving quality of life [12], and has been included in the guidelines for CP/CPPS [13]. Electroacupuncture (EA) is a combination of traditional acupuncture and electrical stimulation, and its advantages include the fact that the stimulus can be controlled and repeated objectively [14]. EA may be more effective than traditional acupuncture in pain management [15, 16]. Studies show that EA is effective for CP/CPPS [17–19]. The waveform is a key parameter of EA. Different waveforms contain different stimulating parameters to generate different clinical effects [20, 21]. However, few studies have described the details of the EA waveform for CP/CPPS [18], which leads to a low evidence level for the clinical recommendation. There is no guidance regarding waveform application, leading to confusion regarding the clinical application. Thus, we designed this study to further evaluate the efficacy of EA and compare the effects of EA with different waveforms to provide reliable evidence and optimize the waveform of EA on CP/CPPS.

## 2. Materials and Methods

### 2.1. Trial Design

This study is a patient- and assessor-blinded, randomized controlled trial. This study was conducted in accordance with the principles of the Declaration of Helsinki [22] and has been approved by the Chinese Ethics Committee of Registering Clinical Trials (ChiECRCT20210053). This trial has been registered on the Chinese Clinical Trial Register (ChiCTR2100044418).

### 2.2. Setting and Participants

Eligible patients were recruited from The Seventh People's Hospital affiliated to the Shanghai University of Traditional Chinese Medicine from 18^th^ March 2021 to 31^st^ January 2022.

Subjects were included if they meet the diagnostic criteria of CP/CPPS according to the National Institutes of Health (NIH) consensus [3], were aged 18–50 years, reported a total score of at least 15 on the National Institutes of Health Chronic Prostatitis Symptom Index (NIH-CPSI), and agreed to participate in this study and sign the informed consent form. We excluded men with other types of prostatitis; history of prostate surgery or invasive treatment; severe heart, liver, kidney, nervous system disease, or mental illness; had a taboo on acupuncture treatment; or failed to cooperate with researchers.

### 2.3. Randomization and Blinding

Subjects were randomly assigned to 3 groups at a ratio of 1 : 1 : 1 by the “Proc Plan” program of SAS 9.4 software (SAS Institute, Cary, NC, USA). The length of the block was set as 6. Opaque sealed envelopes were used to conceal the randomization numbers and the group assignments. Only the acupuncturists have access to the treatment allocation. The patients, outcome assessors, and data analysts will be unaware of the group assignments.

RETRACTED

### 2.4. Interventions

The acupuncture points used in this study are Zhongji (CV3), Guanyuan (CV4), and Dahe (KI12), which are based on our previous study and literature analysis [23, 24]. Patients assume a supine position, and acupuncturists use a 75% alcohol cotton ball to sterilize the skin around the acupoints.

Acupuncturists insert acupuncture needles into the acupuncture point (0.30 × 75 mm, Hwato disposable acupuncture needle, Suzhou Medical Appliance Factory, Suzhou, China). For CV3, CV4, and KI12 (bilateral), the insertion angle is approximately 45°, with the needle tip facing towards the bladder. The insertion depth of the needle is approximately 25–40 mm. After insertion, the acupuncturists gently manipulate (twist) the needle for 1 min to achieve the Deqi sensation (a feeling of soreness, tingling, or bloating) from the patients' local site to the perineum and urethra. Then, the electrode of the EA device (Hwato SDZ-III, Suzhou Medical Appliance Factory, Suzhou, China) was connected to the needle body (the left KI12 + CV4 and the right KI12 + CV3). Then, the acupuncturists set the stimulation parameters: the continuous wave-4 Hz group A's stimulation is 4 Hz; the continuous wave-20 Hz group B's stimulation is 20 Hz; the dilatational wave group's stimulation is 4/20 Hz.

For all three groups, manipulation of the needles by twirling evenly was performed for 1 min in the middle of the treatment period once. The entire treatment procedure took 20 minutes, and patients receive the intervention last for 4 weeks (twice a week), totaling 8 sessions. The treatment frequency was based on a previous study [25]. Relevant drugs or other interventions for CP/CPPS were prohibited during the trial unless patients cannot endure the symptoms.

### 2.5. Measurement and Outcomes

The National Institutes of Health Chronic Prostatitis Symptom Index (NIH-CPSI) was used as the primary outcome measure. NIH-CPSI is a valid, reliable, and widely used questionnaire that aims to evaluate the symptoms of CP/CPPS [26]. It has a total possible score of 43 and contains 9 items that are scored in 3 domains as follows: pain/discomfort (location/type, frequency, and severity, 0–21 points); urinary symptoms (0–10 points); and quality of life (0–12 points). A higher score indicates worse symptoms and vice versa. The severity of CP/CPPS can be graded according to the total scores: mild (1–14), moderate (15–29), or severe (30–43).

RETRACTED

The NIH-CPSI assessment was performed at baseline, week 1, week 2, week 3, week 4, and week 20 (follow-up).

The secondary outcomes include [27] (a) changes in the score of the International Index of Erectile Function 5 (IIEF-5); (b) changes in the Hospital Anxiety and Depression Scale (HADS) score; and (c) changes in the NIH-CPSI response rate. The IIEF-5, HADS, and NIH-CPSI response rate assessments were performed at baseline, week 4, and week 20 (follow-up).

The IIEF-5 is a valid and reliable questionnaire with high sensitivity and specificity for patients with ED [28]. It consists of 5 items, and each of the items is rated from 0 (no intercourse) to 5 (almost always). The total score ranges from 5 to 25, with lower scores indicating more severe ED. The severity of ED can be graded as mild (12–21), moderate (8–11), or severe (0–7).

The HADS is a valid and reliable instrument to screen depression and anxiety and is composed of two subscales, hospital anxiety (HA) and hospital depression (HD) [29]. It includes 14 items, of which 7 items assess anxiety and 7 items assess depression. The severity of anxiety or depression can be graded as negative (0–7), mild (8–10), moderate (11–14), or severe (15–21).

The NIH-CPSI response rate is the percentage of the change in the NIH-CPSI score after treatment ((score after treatment − score before treatment)/score before treatment × 100%).

### 2.6. Adverse Events

Possible adverse reactions to treatment, such as sickness, unbearable needle pain, severe postneedle pain lasting more than 2 hours, local hematoma, and infection; other discomforts (fatigue, palpitation, dizziness, headache, insomnia, or other symptoms); and other unforeseen adverse events were recorded. Due to the low known risk of EA and small sample size [30, 31], the data and safety monitoring committee was not established in this study.

### 2.7. Sample Size

On the basis of previously published data and our study [17], the sample size was calculated by the mean decreased value of the NIH-CPSI score after each type of EA treatment to detect a significant difference between any two groups with a power of 90% and a significance level *α* = 0.05 (two-sided). Considering a 10% dropout rate, the total sample size required was 108 patients with 36 participants in each group.

### 2.8. Statistical Analysis

Continuous data were represented by the mean ± SD, and categorical data were represented by the frequency rate. The changes from baseline in NIH-CPSI among the groups were analyzed by the repeated measure analysis of variance. Demographic data and the change in IIEF-5 and HADS were analyzed by the one-way ANOVA with post hoc multiple comparisons using Tukey's test. The NIH-CPSI response rate and other ratios were analyzed by the chi-square test.

RETRACTED

The data analyses in this study were carried out using the Statistical Package for Social Science software (SPSS version 25.0, IBM Corp, New York). All tests of significance were two-tailed, and a *P* value less than 0.05 was regarded as statistically significant.

## 3. Results

### 3.1. Participant Characteristics

134 participants were screened from 2 sites. After excluding 26 participants, 108 were enrolled. After randomization, 9 participants withdrew their consents, as shown in Figure 1. Baseline characteristics were similar among the three groups, as shown in Table 1.

### 3.2. Efficacy Analyses

At week 4, CP/CPPS response rates were 66.7%, 62.5%, and 88.2% in the 4 Hz, 20 Hz, and 4/20 Hz groups, respectively, as shown in Table 2. The response rate in the 4/20 Hz group was higher than that in the 4 Hz group and 20 Hz group (*P* < 0.05). There was no significant difference in NIH-CPSI total score between the 4 Hz group and the 4/20 Hz group in the period of treatment (*P* > 0.05). From the third week after treatment, the NIH-CPSI score in the 4/20 Hz group was lower than that in the 4 Hz group and the 20 Hz group (*P* < 0.05), as shown in Figure 2. To further study the therapeutic effect of EA with different waveforms on CP/CPPS, we further analyzed the three subscales of NIH-CPSI. After treatment, there was no significant difference in the reduction of pain and discomfort subscales between the 4 Hz group and the 20 Hz group (*P* > 0.05), while the 4/20 Hz group had a higher reduction in pain and discomfort scores compared with the 4 Hz group and the 20 Hz group (*P* < 0.05). There was no significant difference in the reduction degree of urination symptoms and quality of life among the three groups (*P* > 0.05), as shown in Figure 3.

Compared with baseline, the IIEF-5 scores in all three groups were increased (*P* < 0.05). After treatment, there was no significant difference in IIEF-5 scores between the 4 Hz group and the 20 Hz group (*P* > 0.05), while the IIEF-5 score in the 4/20 Hz group was higher than that in the 4 Hz group and the 20 Hz group (*P* < 0.05). Besides, the change in the IIEF-5 score in the 4/20 Hz group was significantly higher when compared with that in the 4 Hz group and 20 Hz group (*P* < 0.05), as shown in Table 2.

The HADS scores in all three groups were decreased (*P* < 0.05). However, there was no significant difference in HADS scores among the three groups (*P* > 0.05), as shown in Table 2.

### 3.3. Safety Analyses

The results show that the adverse events were mild and transient. No serious adverse events were reported in all groups, as shown in Table 3.

RETRACTED

## 4. Discussion

Acupuncture therapy has been shown to have good therapeutic effects on CP/CPPS, which has been recommended by guidelines and the Cochrane systematic review [13, 32]. However, due to insufficient evidence, there is no recommendation for EA parameter application. The waveform is one of the key factors of EA. Different waveforms contain different stimulating parameters to generate different therapeutic effects. However, a few studies do not describe the details of the EA waveform for CP/CPPS [18], which leads to many discrepancies in its application. Considering that different types and parameters of acupuncture may have different potential effects [33], it is necessary to conduct a trial to standardize the EA waveform and improve the level of evidence.

Continuous waves and dilatational waves are the two most common EA waveforms on CP/CPPS. The continuous wave consists of a single pulse waveform, and it can regulate muscle contractions [14]. Studies show that continuous-wave EA can improve the maximum urinary flow rate, mean urinary flow rate, and EMG amplitude of the urethral sphincter and relieve the urethral sphincter and pelvic floor muscle to relieve the symptoms of abnormal urination in patients with CP/CPPS [17, 34]. In addition, low-frequency continuous waves are more suitable for managing chronic pain than high-frequency continuous waves [35]. The dilatational wave is the alternating output waveform of sparse waves and dense waves. It could boost blood circulation and have an antiinflammatory effect [14]. Studies show that dilatational-wave EA has a better analgesic effect, in which the 4/20 Hz waveform has a better analgesic effect on inflammatory pain and could extend the duration of acupuncture sensation (Deqi) [36, 37]. At present, 4/20 Hz is the most widely used dilatational wave parameter in clinical practice. Thus, 4/20 Hz was used in this study.

CP/CPPS main symptoms include urogenital pain, lower urinary tract symptoms, sexual dysfunction, and psychological problems [27]. Therefore, the present study observed not only the effects of electricity on pelvic pain and urination symptoms but also erectile function and anxiety and depression in CP/CPPS patients.

The primary outcome of this study showed that the dilatational-wave EA has a greater NIH-CPSI response rate when compared with the continuous wave. To further analyze the effect of different EA waves on CP/CPPS, the NIH-CPSI subscales in each group were analyzed. Dilatational-wave EA showed better efficacy than continuous waves in the terms of pain and discomfort, while the effect of the two waves of EA on improving urination symptoms and quality of life in CP/CPPS patients was similar. It is assumed that the dilatational wave is better than the continuous wave in the treatment of CP/CPPS, which may be owing to the better improvement of pain and discomfort symptoms. We speculate that it may be on account of the sparse and alternating output of the dilatational wave, which could eliminate inflammatory edema and overcome the deficiency of single wave with adaptation.

RETRACTED

Erectile dysfunction is a common and unaware symptom of CP/CPPS, characterized by the inability of the penis to achieve or maintain an adequate erection, resulting in difficulty in achieving satisfactory sexual performance [38]. The most common etiology of erectile dysfunction in CP/CPPS patients is vascular factors, and the reduction of endothelium-dependent vasodilation due to endothelial dysfunction is an important factor in its occurrence [39]. Honjo et al. observed that acupuncture improved pelvic vein congestion in CP/CPPS patients using ultrasound [40]. The results of this study showed that the dilatational wave is superior to continuous wave for the improvement of erectile dysfunction. The dilatational wave could increase metabolism, promote qi and blood circulation, and improve tissue nutrition, which may be the reason why the dilatational wave showed a better effect.

The most common symptoms of CP/CPPS patients are anxiety and depression [41]. The results of this study indicate that both continuous and dilatational waves could improve patients' anxiety and depression, which may result from the improvement of symptoms and the treatment for mental state. However, different waveforms had similar improvement effects on anxiety and depression, while the trend of HADS scores' reduction of the dilatational wave is higher than that of the continuous wave, which is worthy of further observation.

## 5. Conclusion

To sum up, dilatational and continuous waveforms of EA could both effectively alleviate the symptoms of prostatitis, erectile dysfunction, anxiety, and depression in CP/CPPS patients. The dilatational wave is better than the continuous wave in improving erectile function and pain symptoms of chronic prostatitis, which may be a preferred waveform for CP/CPPS.

## Figures and Tables

**Figure 1:** Flowchart of this study.

**Figure 2:** Mean change in NIH-CPSI total score.

**Figure 3:** Mean change in NIH-CPSI subscales. *Note*. ^*∗*^*P* < 0.05 compared with the 4 Hz group; ^#^*P* < 0.05 compared with the 20 Hz group.

**Table 1:** Participant baseline characteristics.

Characteristics	4 Hz group	20 Hz group	4/20 Hz group
Age (y), mean (SD)	30.00 (6.90)	32.63 (7.88)	31.59 (6.82)
Race, *n* (%)			
Han	30	28	27
Minorities	3	4	7
BMI (kg/m^2^), mean (SD)	21.65 (1.66)	22.17 (2.64)	22.79 (2.66)
Marital status, *n* (%)			
Married	15	17	17
Unmarried	18	15	17
Median sexual frequency per week	1.2	1.5	1.1
Months with CP/CPPS, mean (SD)	15.30 (23.78)	14.41 (24.09)	16.38 (27.53)
Subtypes of CP/CPPS, *n* (%)^&^			
III-A	16	14	16
III-B	13	13	16
Previous treatment, *n* (%)			
Acupuncture	0	0	0
Herbal medicine	2	2	3
Antibiotics	7	6	9
Alpha-blockers	13	14	17
M-receptor blockers	6	3	4
5*α*-reductase inhibitors	2	2	2
NIH-CPSI score, mean (SD)	22.88 (2.60)	23.10 (2.74)	23.59 (2.60)
IIEF-5 score, mean (SD)^^^	14.42 (2.38)	14.68 (1.95)	14.05 (1.65)
HADS score, mean (SD)	15.30 (2.05)	14.84 (2.46)	15.64 (2.43)

^&^Four participants in the 4 Hz group, 5 patients in the 20 Hz group, and 2 patients in the 4/20 Hz group did not complete the examination of prostatic fluid. ^Five participants in the 4 Hz group, 3 patients in the 20 Hz group, and 4 patients in the 4/20 Hz group did not have sex in the last six months. Considering that, their IIEF-5 scores were not included in this study.

RETRACTED

**Table 2:** Primary and secondary outcomes.

Outcome	4 Hz group	20 Hz group	4/20 Hz group
Primary outcome			
Responders, %	66.7	62.5	88.2
Secondary outcomes' change, NIH-CPSI total score			
Wk-1	19.73 (2.65)	20.22 (2.68)	19.47 (2.19)
Wk-2	16.58 (2.80)	17.03 (2.35)	15.56 (1.80)
Wk-3	13.18 (2.32)	13.81 (1.97)	12.03 (1.90)
Wk-4	11.06 (2.08)	11.56 (1.67)	10.09 (1.68)
Change in each domain score of NIH-CPSI at wk-4			
Pain subscale score	5.18 (1.83)	4.94 (1.27)	6.88 (1.41)
Urinary subscale score	3.03 (1.83)	2.84 (1.65)	2.82 (1.99)
Quality-of-life subscale score	3.60 (1.00)	3.75 (1.05)	3.80 (0.98)
Change in IIEF-5 score	4.05 (1.43)	3.90 (1.33)	6.10 (2.12)
Change in HADS score	6.27 (2.05)	6.22 (1.45)	6.85 (1.73)
Patients using other measures	0	1	0

**Table 3:** Adverse events.

	4 Hz	20 Hz	4/20 Hz
Subcutaneous hematoma	3	2	2
Nausea or dizziness	1	0	0
Sharp pain	0	1	0
Abdominal organ injury	0	0	0
Serious adverse	0	0	0

## Data Availability

The simulation experiment data used to support the findings of this study are available from the corresponding author upon request.

## Abbreviations

CP/CPPS: Chronic prostatitis/chronic pelvic pain syndrome
EA: Electroacupuncture
Hz: Hertz (cycles per second)
NIH-CPSI: National Institutes of Health Chronic Prostatitis Symptom Index
IIEF-5: International Index of Erectile Function 5
HADS: Hospital Anxiety and Depression Scale
LUTS: Lower urinary tract symptoms
ANOVA: Analysis of variance
MANOVA: Methods repetitive measure analysis of variance
